# The Role of the Carbohydrate Recognition Domain of Placental Protein 13 (PP13) in Pregnancy Evaluated with Recombinant PP13 and the DelT_221_ PP13 Variant

**DOI:** 10.1371/journal.pone.0102832

**Published:** 2014-07-31

**Authors:** Marei Sammar, Shahar Nisamblatt, Ron Gonen, Berthold Huppertz, Sveinbjorn Gizurarson, George Osol, Hamutal Meiri

**Affiliations:** 1 Prof. Ephraim Katzir Department of Biotechnology Engineering, ORT Braude College, Karmiel, Israel; 2 Department of Obstetrics and Gynecology, Bnai Zion Medical Center, and Technion-Israel Institute of Technology, Haifa, Israel; 3 Institute of Cell Biology, Histology and Embryology/Biobank Graz, Medical University of Graz, Graz, Austria; 4 Faculty of Pharmaceutical Sciences, School of Health Science, University of Iceland, Reykjavik, Iceland; 5 Department of Obstetrics, Gynecology and Reproductive Sciences, University of Vermont College of Medicine, Burlington, Vermont, United States of America; 6 Telemarpe Ltd, Tel Aviv, and Hy-Laboratories, Rehovot, Israel; Medical Faculty, Otto-von-Guericke University Magdeburg, Medical Faculty, Germany

## Abstract

**Introduction:**

Placental protein 13 (PP13), a placenta specific protein, is reduced in the first trimester of pregnancy in women who subsequently develop preeclampsia. A naturally occurring PP13 deletion of thymidine at position 221 (DelT_221_ or truncated variant) is associated with increased frequency of severe preeclampsia. In this study we compared the full length (wildtype) PP13 and the truncated variant.

**Methods:**

Full length PP13 or its DelT_221_ variant were cloned, expressed and purified from E-Coli. Both variants were administrated into pregnant rats at day 8 of pregnancy for slow release (>5 days) through osmotic pumps and rat blood pressure was measured. Animals were sacrificed at day 15 or day 21 and their utero-placental vasculature was examined.

**Results:**

The DelT_221_ variant (11 kDA) lacked exon 4 and a part of exon 3, and is short of 2 amino acids involved in the carbohydrate (CRD) binding of the wildtype (18 kDA). Unlike the wildtype PP13, purification of DelT_221_ variant required special refolding. PP13 specific poly- clonal antibodies recognized both PP13 and DelT_221_ but PP13 specific monoclonal antibodies recognized only the wildtype, indicating the loss of major epitopes. Wildtype PP13 mRNA and its respective proteins were both lower in PE patients compared to normal pregnancies. The DelT_221_ mutant was not found in a large Caucasian cohort. Pregnant rats exposed to wildtype or DelT_221_ PP13 variants had significantly lower blood pressure compared to control. The wildtype but not the DelT_221_ mutant caused extensive vein expansion.

**Conclusion:**

This study revealed the importance of PP13 in regulating blood pressure and expanding the utero-placental vasculature in pregnant rats. PP13 mutant lacking amino acids of the PP13 CRD domain fails to cause vein expansion but did reduce blood pressure. The study provides a basis for replenishing patients at risk for preeclampsia by the full length but not the truncated PP13.

## Introduction

Preeclampsia is a pregnancy disorder that affects about 2–8% of all pregnancies around the globe. According to the WHO preeclampsia remains a major reason for mortality and morbidity of mothers, fetuses and neonates [1]. According to Redman et al. 2008 [2], the disorder comprises new-onset hypertension coupled with damage to the kidney and occasionally to the liver and to the cardiovascular system. Although the etiology of PE is still unclear, it is attributed to multi-factorial causes associated with impaired placentation [3]–[5]. Recent studies have indicated that one of the major causes of placental pathology underlying preeclampsia is the non-homogeneous expansion of the utero-placental vasculature, causing irregular and pulsating blood supply to the placenta, associated with villous disruption and damage [6] that is further exacerbated by the increased impedance of blood flow and the impact of various maternal and placental derived polypeptides and small molecules [4], [5]. Among these factors is Placental Protein 13 (PP13). A meta-analysis by Huppertz et al. 2013 [7] that was based on 18 studies revealed that low levels of this protein are associated with an increased risk to develop preeclampsia.

PP13 was initially isolated by Bohn et al. 1983 [8], who further harvested and purified 56 placental proteins from human placenta at delivery. While the role of many of these proteins was subsequently revealed, the role of PP13, which is specific to the placenta, is still not fully understood.

A full length PP13 cDNA was sequenced, and the sequence of its full length coding protein has been described by Than et al. 1999, 2004 [9], [10] and by Burger et al. 2004 [11]. Molecular modeling and protein analysis by Visegrady et al. 2001 [12] have shown that PP13 mainly appears as a homodimer of 36 kDa, and belongs to the family of the β–galactoside-specific galectins [13]. This group of proteins is characterized by having a carbohydrate recognition domain (CRD) that is highly conserved among the galectin family members [14]. Studies by Than et al. [10], [14]–[15], Huppertz et al. 2008 [16], Grimpel et al. 2011 [17], Balogh et al. 2011 [18], and Kliman et al. 2012 [19] have shown that in the placenta PP13 is mainly found in the syncytiotrophoblast.

PP13 has a very high affinity to sugar residues, particularly the N-acetyl galactosamine of annexin IIa expressed on the surface of the syncytiotrophoblast and its microvillous membrane [7], [10]. Through fucose residues it binds to cytoplasmic proteins, especially to beta/gamma actin [10]. Moreover, PP13 was found to be involved in calcium mobilization [11], [18], interaction with lysophospholipase A [9]–[11], and to induce the release of prostaglandins from cultured trophoblasts [11].

Decreased levels of first trimester maternal blood and placental tissue PP13 protein [7] and of its corresponding mRNA [15], [16], corresponds to later development of preeclampsia. Stalk et al. 2006 [21] from the group of Hillerman in South Africa searched for polymorphisms in the LGALS13 gene encoding for PP13 both in gene libraries and by sequencing with PCR. They were looking for polymorphic variants of PP13 that could account for the reduced mRNA, and potentially for the reduced PP13 protein in women who subsequently developed preeclampsia [22]. Indeed, Gebhardt et al. 2009 [23] have found in certain ethnic groups in South Africa a deletion of thymidine in position 221 of the open reading frame to be expressed in pregnant women from black origin. Having the mutation was associated with early and very severe preeclampsia [23]. The deletion was anticipated to cause a frame shift of the open reading frame and to yield an earlier stop codon, thereby forming a shorter (“truncated”) PP13 lacking the major carbohydrate recognition domain (CRD). Homozygous carriers of this mutation were not detected, and only heterozygous carriers delivered regardless of whether the mutation donor was the father or the mother [23]. Hillerman and Gebhardt thus drew a correlation between the shorter PP13 mRNA and the reduced PP13 mRNA level in preeclampsia [22], [23].

While the role of PP13 in normal development of the placenta and during pregnancy has not been fully revealed yet, Than et al. [14] have shown that PP13 is involved in apoptosis of T-lymphocytes and macrophages. According to Kliman et al. 2011 [19] this process of apoptosis might turn the decidual layer of the placenta receptive to the invading trophoblasts. In in-vitro studies, Than et al. [14] have shown that the truncated protein failed to induce T-cell and macrophage apoptosis, and thus it was concluded that via the CRD molecular region PP13 turns the placenta immune-tolerant to the invading trophoblasts during placentation and that the CRD is essential for this process.

In this study we cloned and expressed the recombinant wild type PP13 and the DelT_221_ variant and characterized the immunochemical and physiological features of both proteins. In a recent study, Gizurarson et al. 2013 [24] have shown that pregnant rodents exposed to PP13 show a reduced blood pressure. In this paper we wanted to investigate whether beyond the immuno-tolerance impact, the CRD has an additional physiological and morphological impact during pregnancy that is associated with preeclampsia.

## Materials and Methods

### Construction and cloning of PP13 variants

The novel coding variant identified in exon three of the LGALS13 gene represents a deletion of a single thymidine base at nucleotide position 221, resulting in substitution of a leucine with a tryptophan residue at amino acid position 74. The result is a disruption of the open reading frame leading to the production of an earlier stop codon and a truncated protein. The truncation removes 37 amino acids corresponding to part of LGALS13 exon three, and the entire exon 4. The anticipated molecule was profiled (Figure 1) and the area of the naturally occurring mutation was marked.

**Figure 1:** Design of the truncated PP13. Top right insert - the exon and intron organization of PP13 DNA (LGALS13 or galectin 13) showing the 5 and 3 prime ends. The 4 exons are colored black (exon 1), blue (exon 2), orange (exon 3) and brown (exon 4). Figure body - the amino acid sequence of the anticipated protein with amino acid colored according to the respective exons. Red colored – the methionine added to the his tag. The sequences of the wild type recombinant PP13 (rPP13) (top line in each couple sequences) is constructed of 164 amino acids that are aligned with the sequence of the DelT_221_ (Truncated) (the lower of each couple), made of 98 amino acids. First line couple - the his-tag added to the N-terminal followed by the sequences of the first short exon (black), second exon (blue) and a part of the third exon (orange), which are identical in both molecules. Second line couple - continuation of exon 3 (orange) and beginning of exon 4 (brown) for the wild type and for the truncated variant lacking 28 amino acids of exon 3 and 7 amino acids of exon 4. Third line – the rest of exon 4 of the wild type, which is completely missing in the truncated variant (31 amino acids) and the C terminal tail, which is identical in both molecules.

### Cloning and construction of PP13 mutant gene and expression and purification of recombinant truncated PP13 protein

The full length of PP13 wild type was previously cloned in pQE30 plasmid [9]–[11] and was used as a template to amplify the wild type PP13 and its DelT_221_ PP13 mutant (referred to as truncated) sequence by PCR. Two primers were designed with the following sequences: a sense primer: CGAATCCATGTCTTCTTTACCCGTGC and an anti-sense primer: TAAGTCGAGCTCCATCCATATCCCAAACTCAC.

The restriction site sequences of BamH I and Sac I were introduced in the sense and anti-sense primers, respectively. Both primers were synthesized by Sigma-Genosys.

To amplify the truncated PP13 DNA sequence, 1 ng of wild type PP13 DNA was used as a template. 0.1 µM of the above mentioned specific primers, 1 U of plaque forming unit (Pfu) DNA polymerase (Promega, USA), 200 µM deoxyribonucleotide (dNTP)-mix and Pfu DNA polymerase X10 buffer. PCR was carried out at the following temperature cycles: 94°C for 2 min, 94°C for 30 sec, 60°C for 30 sec and 72°C for 1 min over 35 cycles. A final extension was carried out at 72°C for 4 min and the PCR product, analyzed by agarose gel and revealing the expected size of 288 bp, was stored at 4°C until use.

Basically, the procedure for expression of recombinant wild type and truncated PP13 in *Escherichia coli* M15 strain host cells was performed according to the procedure of QIA express (Qiagen, USA) using the expression vector pQE-30 as described by the manufacturer. The PCR product of PP13 DNA was purified by QIAquick PCR purification kit prior to ligation. Both the pQE-30 and the purified PCR product DNA were digested with BamH I and Sac I (New England Biolabs, USA). The digested truncated PP13 insert was ligated into the digested pQE-30 expression vector using T4 ligase (NEB, UK) for 2 h at 22°C. The *E. coli* M15 strain containing the repressor (pREP4) plasmid was transformed with the ligated product and cells were grown on ampicillin and kanamycin selective agar. Positive clones were selected and confirmed by sequence analysis using a pQE sequencing primer (Qiagen, USA). The transfected *E. coli* cells were grown to an *A*600 of 0.9 and isopropyl-β-D-thiogalactopyranoside (IPTG) was then added to a final concentration of 1 mM. The cells were grown for an additional period of 4 h, pelleted for 20 min at 4000 *g*, and stored at −80°C until use. Aliquots were tested by SDS-PAGE to determine the molecular weight of recombinant proteins.

The cell pellet was thawed and resuspended in lysis buffer containing 20 mM Tris-HCl, pH 8, 150 mM NaCl, 5 mM imadizole, protease inhibitor (Roche) and 10% glycerol. The cells were disrupted by applying pressure of 1000 PSi in minicell French press (Thermo, USA). Soluble proteins and the insoluble fraction (inclusion bodies) in the pellet were analyzed. Based on SDS-PAGE analysis, the recombinant wild type PP13 was localized in the soluble fraction, whereas the recombinant truncated PP13 was localized in the inclusion bodies. For purification of wild type PP13, the soluble fraction was filtered through 0.25 µm pore size filters and mixed with 1 ml of pre-equilibrated Ni-NTA agarose (Qiagen) for 1 h at RT. First the Ni-NTA agarose column was washed with 20 ml of wash buffer (20 mM Tris-HCl, pH 8.0, 300 mM NaCl, 20 mM Imidazole, PMSF, Complete and 10% glycerol). Bound recombinant PP13 was eluted with 15 fractions of 1 ml of elution buffer (20 mM Tris-HCl, pH 8.0, 300 mM NaCl, 0.5 M Imidazole, PMSF, Complete and 10% glycerol). PP13 was analyzed by SDS-PAGE (10%). Positive fractions were combined, dialyzed against TBS (20 mM Tris-HCl, pH-8, 150 mM NaCl) and stored at −80°C until use.

For purification and renaturation of truncated PP13, pellets containing the inclusion bodies (0.75 g) were resuspended in binding buffer (20 mM Tris-HCl, pH 8.0, 300 mM NaCl, 5 mM Imidazole, 6 M urea, PMSF, Complete, 1 mM DTT and 10% glycerol). After 1 h of incubation at room temperature, the insoluble proteins were discarded by centrifugation at 20,000 *g* for 20 min. The soluble fraction was filtered through 0.45 µm pore size filters and mixed with 1 ml of pre-equilibrated Ni-NTA agarose (Qiagen) for 1 h at RT. The refolding of the bound recombinant truncated PP13 was performed on the column using a step-wise linear 6 to 0 M urea gradient. First the Ni-NTA agarose column was washed with 10 ml of wash buffer (20 mM Tris-HCl, pH 8.0, 300 mM NaCl, 20 mM Imidazole, 6 M urea, PMSF, Complete, 1 mM DTT and 10% glycerol) followed by washing the column with 10 ml of refolding buffers (wash buffer containing 4, 2, 1, 0.5 and 0 M urea). Bound recombinant PP13 was eluted with 5 ml of elution buffer (20 mM Tris-HCl, pH 8.0, 300 mM NaCl, 0.5 M Imidazole, PMSF, Complete, 1 mM DTT and 10% glycerol). Recombinant, truncated PP13 protein was dialyzed against TBS (20 mM Tris-HCl, pH-8, 150 mM NaCl) and diluted with equal volume of 60% glycerol in TBS and stored at −80°C until use.

### Polyclonal and monoclonal antibodies to PP13

Polyclonal antibodies against PP13 were produced by Interchim (France). Briefly, two rabbits were immunized with 200 µg recombinant His PP13 in complete Freund’s adjuvant followed by four booster injections with the antigen in incomplete Freund’s adjuvant at two weeks interval. Rabbits were bled and antiserum was stored at −20°C. Immunoglobulin fraction (IgG) was purified from the antiserum by protein-A affinity chromatography.

The monoclonal antibodies of lines 27-2-3 and 215-28-3 (each IgG1) were those isolated after mice immunization with the native PP13 isolated from placenta [4] and are the ones used in the ELISA and Delfia PP13 kits as summarized in the meta-analysis [12].

### Gel electrophoresis, Western blot, ELISA and Dot-Blot analysis

The recombinant wild type and truncated PP13 proteins were characterized by SDS-PAGE, Western blot and ELISA analyses. Truncated PP13 was resuspended in Laemmli sample buffer, loaded and separated by 15% SDS- polyacrylamide gel electrophoresis (PAGE) under reducing and non-reducing conditions. Protein profile was visualized by staining the gel with Gel-Code dye (Pierce).

For Western blot analysis, recombinant PP13 proteins subjected to SDS-PAGE were electro-transferred to nitrocellulose membrane. After blocking non-specific binding sites with 5% non-fat milk in 20 mM Tris/HCl buffer at pH 8.0 supplemented with 150 mM NaCl, the blots were incubated with primary anti-PP13 antibodies (mAbs and pAbs) overnight at 4°C, followed by peroxidase-conjugated secondary antibody (Jackson ImmunoResearch Laboratories, USA). Antigen antibody complex was detected by enhanced chemiluminescence system-ECL (Biological industries, Israel).

Enzyme-linked immunosorbent assay (ELISA) was used to test the reactivity of anti-histidine, anti-PP13 monoclonal antibodies (mAbs) and anti-PP13 polyclonal antibodies (pAbs) with recombinant PP13 proteins. Briefly, flat bottom ELISA plates (Nunc, USA) were coated with 250 ng affinity purified recombinant PP13 (rPP13) per well overnight at 4°C followed by blocking non-specific sites with 1% bovine serum albumin (BSA, Sigma, Israel) in phosphate-buffered saline (PBS), pH 7.4. The plates were then incubated with serial dilutions of mouse anti Histidine mAbs or anti-PP13 mAbs and isotype-matched negative control antibody or rabbit anti-PP13 pAbs or matched pre-immune IgG for 2 h at room temperature (RT). The bound antibodies were then marked by 2 h incubation with goat anti-mouse IgG (mAbs) or goat anti-rabbit (pAbs) conjugated to horse radish peroxidase (HRP). Extensive washing with PBS containing 0.05% Tween was performed between steps. The reaction product was developed with 3,3′,5,5′-tetramethylbenzidine (TMB, Dako, Denmark), stopped with 2 N HCl, and the optical density was measured by ELISA reader (Tecan Sunrise absorbance reader for microplates, Neotech Ltd., Kfar Sabba, Israel) at 450 vs 650 nm.

To conduct Dot blot analysis wild type and truncated PP13 were absorbed to nitrocellulose membrane (Biorad, Israel) and free binding sites were blocked with 5% milk in Tris buffered saline pH 8.0 (TBS) for 1 h. Membrane was incubated with anti PP13 antibodies for 2 h at 37°C and free antibodies were washed with TBS-Tween 20. To detect bound anti-PP13 antibodies, a secondary antibody conjugated to HRP enzyme was added to the membrane and incubated for 60 min at RT followed by discarding the free excess antibodies by washes as indicated above. Enhanced chemiluminescene (ECL) reagents were used as a substrate for the HRP and the signals were visualized, captured and analyzed by using the LAS3000 image system (Fuji, Japan).

### Clinical cohorts

Ethical committees at Bnai-Zion Medical Center, Haifa, Israel approved the two cohorts of the study. Patients provided individually signed written informed consent to use their specimen and all personal details were anonymized. All informed consents were stored in a locked cabinet along with the source data as required by Israel Ministry of Health. The study was conducted according to principles of GCP, patient safety and privacy, as guided by the Bnai Zion’s Ethics Committee. The Israeli cohorts were already described in the past [17], [20], [25]. The longitudinal assessment of this large first trimester cohort was already described by Than et al. 2011 [25] and consists of 1078 women who attended first trimester assessment of pregnancy disorders of which 20 developed preeclampsia. A subgroup of 56 women of this cohort was admitted to social termination during the first period of pregnancy, and these women (excluded from the analysis of the large cohort described in ref 25] provided placental specimens in addition to blood and urine samples [17]. A sub-group of the large cohort admitted for delivery at GA 26–40 weeks provided not only blood samples but also placental samples, amniotic fluid and fetal umbilical cord blood [17], [20]. This sub-cohort included14 subjects who developed preeclampsia (as defined in [27]), with 7 cases delivered before GA 35, 10 cases of iatrogenic preterm delivery [26] who delivered before 35 weeks, 3 cases of IUGR who delivered at GA <35, and 107 normal term deliveries (GA≥37).

Severe preeclampsia was determined according to the world congress for the study of hypertension disorders in pregnancy [27] and according to the American College of Obstetrics and Gynecology and the American Society for the Maternal and Fetal Medicine [28], [29]. The definition includes hypertension developing after 20 weeks in patients having systolic blood pressure (SBP)≥160 mm Hg or diastolic blood pressure (DBP)≥110 mm Hg coupled with proteinuria of 3+ at dipstick or >300 g/dl per 24 h urine collection.

### Animal Experiments

Animal Research committee of the University of Vermont, College of Medicine approved the study in pregnant rat in compliance with the 3R principles of ethics. Female Sprague-Dawley rats (12 weeks old), purchased from Charles River Laboratories (Wilmington, USA), were housed in metabolic cages and allowed to acclimate in the Small Animal Facility at the University of Vermont, College of Medicine, for 72 h prior to use. They were then mated by a male, and their pregnancy was verified by the presence of a seminal plug. Each was then instrumented according to Osol and Moore 2014 [30] with 2 ml Alzet osmotic pumps (Alzet, CA, USA) surgically implanted subcutaneously into the periscapular region. The pumps were implanted at gestational day 8 after loading with 127 ng rPP13 (n = 9), the DelT_221_ variant (n = 6) or saline (n = 6). As described by Gizurarson et al. 2013 [24] the pumps released approximately 0.625 ng PP13/h over 5–7 days (term = day 22).

Blood pressure and heart rate were measured prior to implantation of the osmotic pumps on gestational day 8 and then on gestational days 10, 13 and 15 using a tail cuff oscillometric blood pressure system (Coda Kent Scientific Corp, CT, USA). The animals were allowed to acclimatize in the measurement chambers for about 30 min prior to the initiation of measurement.

### Uterine vasculature

Each animal was euthanized with an intra-peritoneal injection of Nembutal on day 15 or day 21 of gestation, followed by decapitation, laparotomy, and dissection of the uterus and its vasculature. The entire uterus, including placentas and pups was pinned in a Petri dish coated with silicone (SilGard). The petri dish was filled with regular 10 mM HEPES saline at 4°C that contained a mixture of papaverine (10^−4^ M) and diltiazem (10^−6^ M) to assure complete relaxation. Each horn of the rat uterus and its vascular arcade were photographed with a calibrated stereomicroscope (Zeiss, Germany) to measure the uterine vein inner diameter. Three measurements were made along the length of each vein and averaged to provide one value per animal.

### Statistical Analysis

Baseline and delivery characteristics were compared between cases and controls using Fisher’s exact test for categorical variables and Wilcoxon Rank Sum test for continuous variables. PP13 blood level and amount released to culture medium were compared after converting blood level to gestational week specific multiple of the medians (MoM) further adjusted to body mass index (BMI) [17], [20], [25]. Scattered analysis and T-test were used to compare the PP13 level in normal pregnancy and placental disorders. All *P* values were two-tailed. P<0.05 was considered significant.

## Results

### Cloning, expression and purification of recombinant PP13 variants

Results obtained from small-scale expression cultures of His-tagged truncated PP13 indicated that an IPTG induction period of 4 h was the optimal timing for inducing PP13 expression for both wild type and truncated PP13 (not shown). As shown in Figure 2A the majority of His-tagged truncated PP13 protein of an apparent molecular weight of 12 kDa was found in inclusion bodies (pellet), while the wild type PP13 was revealed in the soluble fraction (supernatant). Accordingly, both proteins were purified by Ni-NTA matrix under native or denaturing conditions. For purification of truncated PP13, inclusion bodies were solubilized by a strong denaturant (urea) to allow binding to Ni-NTA followed by renaturation and refolding by sequential washes of decreasing concentrations of urea (6 M to 0 M urea) prior to elution as shown in Figure 2A. Accordingly, the purified samples separated with SDS-PAGE in reducing conditions yielded a ∼18 kDa molecule corresponding to the “wild type” recombinant rPP13 monomer and a ∼12 kDa protein corresponding to the truncated variant (Figure 2B). Sequence analysis, amino acid analysis and ion residue analysis confirmed the corresponding results: 164 amino acids (AA) with C_846_H_1287_N_231_O_238_S_10_ for rPP13 and 98AA with C_495_H_754_N_144_O_137_S_6_ for the DelT_221_ variant (Figure 1).

**Figure 2:** Purification and detection of the wild type and the truncated PP13. A - Purification and characterization of heterologously expressed His-tagged truncated PP13. Expression of 6 His-tagged PP13 in *E. coli* was induced by IPTG. The protein was purified on Ni–NTA–agarose under denaturing conditions and separated on 15% SDS–PAGE. The total proteins were visualized by Gel Code blue staining. CL-clear lysate, Pel-cell pellet, Sup-Supernatant, FT-Flow through, W1 - 6 M urea, W2–4 M urea, W3 - without urea. B - The combined eluted fractions were separated by SDS-PAGE and stained by Gel-Code blue and the wildtype and truncated protein are shown. C - Proteins were electrotransferred by Western-blot. Only the His-tagged wild type (lane-1) but not the truncated PP13 (lane-2) was detected with the ELISA capture mAb (mAb1) and the detecting mAb (mAb2) as revealed with marking by HRP-conjugated rabbit anti mouse IgG and ECL detection reagent.

### Biochemical characterization of recombinant PP13 variants

As shown in Figure 2C, in Western blots the PP13 specific monoclonal antibodies (mAbs) recognized only the wild type PP13 but neither mAb 27-2-3 (1^st^ mAb) nor mAb 215-28-3 (2^nd^ mAb) recognized the truncated variant. To further understand the lack of recognition, a Dot Blot analysis was performed assuming the 3D configuration is better preserved by this semi-analytical method. However, the Dot Blot analysis revealed that the mAbs exert excellent recognition of the wild type dot but failed to recognize the truncated variant either completely (2^nd^ mAb) or recognized it only very lightly (1^st^ mAb, Figure 3A). On the contrary, incubation with rabbit polyclonal antibodies (pAbs) revealed a very strong reactivity of either the wild type PP13 or the truncated variant (Figure 3B) with a slowly fading signal still detecting up to 230 pg of the DelT_221_ variant compared to normal rabbit serum or HRP controls. The pAbs recognized PP13 down to a concentration of 675 pg (wild type) and 232 pg (truncated) per dot. All other panels were negative (Figure 3B).

**Figure 3:** Dot blots. A – Both 1^st^ and 2^nd^ mAbs recognize the wild type PP13 over background at 10 ng/ml (top panel). Using the same conditions the 1^st^ mAb barely recognizes the truncated PP13 and the 2^nd^ mAb doe’s not show a signal at all. B – Serial concentration of the wild type and truncated PP13 variants were placed on nitrocellulose, reacted with rabbit polyclonal antibodies to PP13 (pAbs) (top panel), or non-immune serum (NRS, middle panel) or without antibodies (HRP negative control) and reacted with goat anti rabbit IgG conjugated to HRP.

Further Western blots revealed a very specific recognition of both the truncated and the wild type PP13 by the rabbit pAbs in both reduced and non-reduced conditions compared to pre-immune rabbit serum or HRP (Figure 4). The pAbs also recognized the native PP13 purified from the placenta (Figure 4). The latter is also recognized by each of the mAbs as was previously demonstrated [10], [11], [15], [20]. Comparison of reduced and non-reduced conditions showed that under non-reduced conditions the pAbs also recognized dimers, trimers, tetramers and polymers of wild type PP13 (Figure 4A). Under the experimental conditions, no polymerization of the truncated or the native protein could be identified in the non-reduced conditions although the latter is known to be stable in human blood as a dimer [9]–[11].

**Figure 4:** Western blots with polyclonal pAbs. The recombinant (rPP13) wild type PP13, its truncated variant (DelT_221_) and the native molecule (nPP13) purified from the placenta were separated by 15% SDS PAGE under non-reducing (A) or reducing (B) conditions, electro transferred to nitrocellulose and reacted with rabbit pAbs to PP13 (J67), pre-immune rabbit IgG (Jo) or without antibody (HRP negative control) followed by incubation with goat anti rabbit IgG conjugated with HRP. A single band is shown for the native and truncated PP13 in both reduced and non-reduced conditions. The recombinant wild type generates a single band in reduced conditions but in non-reduced conditions dimer, trimer and tetramer PP13 are revealed. The recombinant PP13 is heavier than the native protein due to the his-tag and extra tail sequence in the recombinant protein.

The pAbs reacted with both wild type and truncated PP13 in a dose dependent manner as shown in Figure 5A, whereas no reactivity was seen with the control NRS. The pAbs recognized the wild type PP13 at a concentration of 20 pg and each of the mAbs (Figure 5B) recognized the wild type PP13 at a concentration of 1 and 3 pg for mAb 27-2-3 and 215-28-3, respectively. The polyclonal antibodies also recognized the truncated PP13 (Figure 5A) at a concentration of 0.5 ng but none of the mAbs recognized the truncated PP13 (Figure 5B). Anti-histidine antibodies were used as a positive indication that both PP13 and the truncated variant were indeed bound to the wells of the ELISA microplates (Figure 5B). The 50% reactivity of pAb was at 1∶5000 and 1∶10000 for truncated and wild type PP13, respectively.

**Figure 5:** Capture ELISA. Plates were coated with the wild type PP13 or the truncated variants at 2.5 µg/ml, blocked with 1% BSA in PBS and then incubated with serial dilutions of pAbs (A) or of the 1^st^, 2^nd^ and anti Histidine mAbs followed by development with goat ant rabbit (A) or anti mouse (B) IgG conjugated to HRP. 5A – The signal is gradually reduced over a log dilution of the antibody concentration with either the wild type (diamonds, purple) or truncated (circles, blue) PP13 variant compared to the pre-immune response (diamonds and circles, respective colors). 5B – Both first (top panel) and second mAbs (middle panel) recognized the wild type PP13 (blue) but not the truncated (red) protein. Antibodies to the His-Tag (bottom panel) recognized both of the proteins.

In sandwich ELISA performed in the regular or the inverted version, the analytically detected concentration of rPP13 by the mAbs was 7 and 9 pg/ml but none of the mAbs recognized the truncated PP13 (not shown). Taken together the results indicated that the mAbs are not able to identify the DelT_221_ variant with their specific binding epitopes.

### Animal Studies

#### Blood pressure

As we have reported for IV PP13 injection [24], the continuous release of wild type rPP13 into rats was followed by reduction of the rats’ blood pressure with mean arterial blood pressure (MAP) reduction from 100 mm Hg before exposure to 75 mm Hg and 80 mm Hg with the wild type and DelT_221_, respectively (Figure 6A) (p<0.0001 for each compared to saline control). With the wild type, the reduced blood pressure reurn to normal in 15 while with the DelT_221_ variant the effect appeared to recover faster, reaching normal level approximately 2 days earlier (Figure 6). While recovery was faster after the exposure to the truncated mutant, it appeared that the reduction in blood pressure following exposure to PP13 did not require the integrity of the full PP13 molecule including the carbohydrate recognition domain (CRD).

**Figure 6:** Studies in pregnant rats. A. Mean arterial pressure (MAP) of pregnant rats after sub cutaneous implantation of slow releasing osmotic pumps with PP13 (black bars) (n = 9), the DelT_221_ mutant PP13 (dark gray bars) (n = 6) or saline (light gray bars) (n = 6). Mean values ± SD of MAP are presented from day 8 (before pump implantation), and after implantation on days 10, 13 and 15 of gestation (2, 5 and 7 days after pump implantation). P values show significances between saline controls and PP13 and saline controls and DelT_221_. B. The main uterine vein diameters of pregnant rats after pumps implantation is shown for 4 rats in each of the PP13 group (black bars), the DelT_221_ mutant group (dark gray bars) or saline control group (light gray bars). Mean values ± SD of the main uterine veins are presented for the 21^st^ day of gestation (e.g. –9 days after the pumps were emptied from their releasing material). P values show significances compared to the saline control group and the DelT_221_ mutant group.

#### Uterine Vein expansion

The utero-placental vasculature underwent structural arterial expansion as tested at gestational day 21 (Figure 6B). Administration of PP13 beginning on day 8 of pregnancy induced a significant (50%) increase in uterine vein diameter relative to controls. This effect was not apparent in rats that received the DelT_221_ variant (Figure 6B).

### Patient Samples

As published earlier, in the cohort from Israel, we were able to detect reduced blood levels of the PP13 protein in the first trimester in 85% of the cases and 15% of the controls [25], and also found reduced PP13 RNA in the placenta of all preeclampsia cases near the time of delivery [20], and in 30% in the first trimester (Sammar et al., unpublished results). However, in this large Israeli cohort (PE and unaffected cases) the DelT_221_ mutation was not found with PCR amplification of placental tissue or blood samples or by immune precipitation of placental tissue (data not shown). This indicates that the decreased blood PP13 and decreased placental PP13 mRNA cannot be accounted for by having the DelT_221_ mutation.

## Discussion

### Main study finding

The main findings of this paper are as follows: (1) We report the successful cloning, expression, production, purification and characterization of the wild type recombinant PP13 and its DelT_221_ variant, the latter corresponding to a naturally occurring mutation among black people in South Africa associated with high frequency of severe preeclampsia. The DelT_221_ variant is a shorter molecular variant lacking the carbohydrate recognition domain on exon 4 and part of exon 3. (2) The primary structural change of DelT_221_ is also associated with protein misfolding and its routing into inclusion bodies. Implications for short life span of the DelT_221_ variant in the placenta are further discussed below. (3) The truncated variant is recognized by polyclonal antibodies to PP13 using Dot Blots, Western blots and ELISA. On the contrary, the truncated variant is not recognized by two PP13 specific mAbs indicating the epitopes of these mAbs are missing in the truncated variant or are not available due to misfolding. (4) Both, truncated and wild type PP13 caused blood pressure reduction in pregnant rats. (5) Wild type PP13 supplementation during pregnancy induced expansion of the utero-placental vasculature in rats, while the effect was not present with the truncated variant. (6) The deletion mutation of thymidine in position 221 of the open reading frame accounting for the truncated DelT_221_ variant was not found among the Caucasian population in Israel, although we did determined reduced first trimester PP13 in 80% of the preeclampsia cases who also had reduced placental PP13 mRNA.

### Shorter Version of PP13

Gebhardt et al. 2009 [23] have discovered the naturally occurring DelT_221_ variant of PP13 and have identified its higher frequency among early onset preeclampsia cases in women from black and colored origin in South Africa. No homozygous variant of the DelT_221_ was detected in the course of the study suggesting that DelT_221_ homozygosity may be incompatible with life. In South Africa the mutation was found in 8 mothers of the 338 control patients (2.4%) and 6 mothers of the 35 preeclampsia cases (17.1%) [23]. Additional analysis (unpublished data kindly provided by Hillerman and Gebhardt) compared the mutation in the newborns and found that it appeared in only 4 cases of the controls (1.8%) and 8 PE cases (22.9%). As the DNA of the placenta and of the newborn are the same, it appeared that regardless of the origin of the gene donor (maternal or paternal), there was a significant increase in the frequency of the mutation in preeclampsia cases in the black and colored population in South Africa. The newborn statistics indicated a 10-fold increase in the mutation frequency in the PE group compared to control. The Odds ratio was 7.2∶1 when calculated from the mother having the mutation and 12.5∶1 when calculated from the newborn/placenta, indicating the additional paternal contribution to mutation carriers among the off-springs.

Here we studied a recombinant variant of PP13 that was constructed according to this mutation. The thymidine deletion in position 221 is associated with a frame shift in the open reading frame and the formation of an earlier stop codon. The resulting protein has a molecular weight of 11 kD compared to 18 kD of the wild type. The human DNA polymorphism as expressed in the DelT_221_ mutation was not identified so far in the Caucasian population of quite a large cohort in Israel. At present it remains to be seen whether having only one locus producing wild type PP13, while the other being rapidly degraded, is associated with having low blood levels of PP13 in comparison to the situation of having both loci generating wild type PP13. Such a study has to be conducted in Africa. However, it is tempting to speculate that having not any locus generating wild type PP13 is associated with very early pregnancy loss, missed abortion or infertility.

### Misfolded protein

Already in E. coli, the expressed DelT_221_ protein was routed into inclusion bodies, a phenomenon that was previously reported in relation to the expression of misfolded proteins by Kraft et al. 2010 [31] and by Gerrec et al. 2013 [32]. It appears that the bacteria “conceived” the truncated protein variant as “junk” and therefore removed it by routing it into the inclusion bodies. High concentrations of urea were used to refold the protein in bacteria, and recover it out of the inclusion bodies to enable its purification. It remains to be seen what the degradation process of the mutated protein is in human placenta and how to gain its recovery in human with a potential procedure for pH changes [32] or the formation of multi-vascular bodies as described by Wang et al. 2011 [33]. At present we assume that the cytoplasm recognized the misfolded mutated DelT_221_ at a “control checkpoint” already at the endoplasmic reticulum or the Golgi and routes it for a fast turnover to avoid potential toxic effects. This process will prohibit the recovery of this protein variant from mutation carriers unless special biochemical procedures are implemented [31], [33]. Developing such recovery methods seems important to follow the life cycle of the truncated variant in human; given the homozygous DelT_221_ may not be viable. Thus, a special procedure has to be developed to be able to identify the shorter protein version among mutation carriers.

### PP13 Expression in Bacteria

While PP13 is expressed in human and in human like monkey, its expression in bacteria appears to be suitable given that *the PP13 molecule was shown by Bohn et al [8] to have only 0.6% carbohydrate. Therefore, PP13 expression in bacteria, yeast, baculo virus or hamster ovarian cells is not anticipated to generate any difference in term of the final product.*

### Carbohydrate binding

A truncated mutation of PP13 different from the one described here was described by Than et al [14]. The carbohydrate recognition domain (CRD) is consisted of 8 Amino acids (AA) residues, of which 4 AA residues (located on position 53, 65, 72 and 75) form a “pocket” fitting the sugar residue as a key and a lock. Additional 4 AA residues (located in position 55, 57, 63 and 77) add to the affinity to sugar residues. It was already mentioned that the DelT_221_ was identified in the black minority in S. Africa [23]. It lacks only 2AA residues (in position 72 and 75) of the 8 required for the functional CRD, but it i so misfolded that it lost it sugar binding.

The truncated mutation of Than et al [14] has only 55 AA residues resulted of 163 C to T SNP that was identified on a chromosome psuedoPP13 gene and was shown to lack both CRD function and the ability to induce T-Cell apoptosis [14].

### Decreased blood pressure and uterine arterial expansion

One of the physiological effects of PP13 found here in pregnant and non-pregnant rats [also in Ref. 24], is the reduction of blood pressure. This effect seems to be mediated by exon 1 and 2 of the molecule and is unrelated to having or lacking the major CRD since the truncated protein can also cause reduced blood pressure. The extent and duration of the PP13-induced hypotension caused by the mutant compared to the wild type is reduced, which appears to be most likely attributed to the misfolding of the DelT_221_ protein.

Earlier reports indicated that PP13 has an intrinsic phospholipase C activity [9]–[11], and the ability to release prostaglandins [11], thereby causing vasodilation that can presumably reduce blood pressure. Considering exon 1 is very short, the prime molecular region that is the candidate for causing blood pressure reduction is exon 2 [7]. A subsequent study with PP13 mutated variants lacking exon 2 [7] may be useful in shedding light on this part.

The uterine vein morphometric data clearly showed a positive effect of PP13 on uterine vein gestational expansion through mechanisms that remained to be determined, as uterine vein diameters were almost 50% larger in animals infused with PP13 protein (Figure 6B). Notably, this represents true vein growth and in relaxing solution that contained papaverine and diltiazem. Unlike the native protein, which augmented structural enlargement of the main uterine vein, the truncated mutation was without effect (Figure 6B).

It was already discovered that in the human PP13, which is exclusively expressed in the placenta, can be detected in maternal serum as early as 6 weeks of gestation [16]. This period occur after the evolvement of the synsytiotrophoblast where Pp13 is expressed in the placenta. The meta-analysis of all clinical studies has shown that decreased PP13 in maternal blood starts at 6 to 8 weeks of gestation and extends throughout the first trimester in women who will subsequently develop preeclampsia [7], [16], [25]. Thus, the importance of PP13 in the maternal circulation appears relevant to the normal course of pregnancy whether supplied artificially (as in the animal studies described hereby) or whether arrived from the placenta (in human pregnancy). Kliman et al [19] revealed that there is a deposition of PP13 in special zones of necrosis outside the alveioli indicating the large effect of Pp13 is anticipated in the smaller vein. This is now analyzed in our next study where we assess the impact of PP13 on 4 level of the veins and infact found the larger impact on the thinner arterioli.

### Truncation and the increased risk for preeclampsia

The truncated mutation seems to be associated with a 10-fold increased risk to develop preeclampsia compared to control in colored and black populations in South Africa [23]. The homozygous variant was never found indicating this variant may not be vital. Accordingly, having a full length PP13, at least in the heterozygous form, seems enough for a successful pregnancy. The mutation has not been resolved so far in either human plasma, white blood cells or in the placenta among the Caucasian population. A challenging study now uses next generation sequencing and advanced PCR to resolve this mutation at the RNA level during pregnancy among Caucasians using a very large cohort that also includes many African-Caribbean patients in Europe.

### DelT_221_ DNA mutation, reduced PP13 RNA, lower protein level

PP13 is specifically expressed in the placenta [9], [14], [16] and can be detected by immunolabeling mainly in the apical membrane of the syncytiotrophoblast [10], [11], [14]–[18]. Other studies from our group [15], [20] have reported reduced PP13 mRNA in the placenta in preeclampsia, particularly in early and preterm cases. Three different studies have shown reduced PP13 mRNA in chorionic villous sampling in the first trimester and in first trimester blood of patients who subsequently developed preeclampsia [34]–[36]. Accordingly, reduced expression of PP13 is considered as one of the earliest indications for the risk to develop preeclampsia. The use of this approach in testing maternal blood mRNA has yielded a detection rate of 30–50% for a 10% false positive rate, which may be improved with the advance offered by new mRNA isolation and deep sequencing methods also including the identification of mutants such as the DelT_221_ variant.

There are 18 studies today that in a meta-analysis indicated that lower first trimester serum PP13 is associated with an increased risk of preeclampsia [7]. The current study emphasizes the pathway of primary sequence DNA mutation→lower PP13 mRNA→lower protein and its relevance to the development of high risk for preeclampsia. However, the reverse path of low PP13 protein→low PP13 mRNA→DNA mutation failed at the final step. The ways PP13 (or a reduced PP13 level) is involved in preeclampsia varies and one mutation in one part of the PP13 molecule (the CRD domain) cannot provide the complete picture and does not account for the pluripotent origin of preeclampsia and the broad aspects of the disorder. Nonetheless, the study emphasizes new aspects for the role of PP13 and its CRD regulatory domain in pregnancy and preeclampsia.

### PP13 and the changes in the vasculature

According to Kliman et al [19] in human placenta first trimester PP13 is mainly present in the syncytiotrophoblast facing the maternal side from which it is liberated into the veins and the maternal circulation. This PP13 also cross the vein wall (presumably through the intrinsic lysophospholipase activity), and crystalize outside at the “Zones of Necrosis” that are infiltrated by proinflamatory immune cells, that are undergoing apoptosis as was also revealed by Than et al [14]. In cases of low maternal blood PP13 the zones were small or absent and accompanied by impaired spiral artery remodeling. Accordingly, Kliman et al [19] proposed the “diversion” of PP13 acting as a decoy inflammatory signal.

In this study *PP13 (but not its truncated mutant) causes a significant expansion of the veins in the utero-placental vasculature in the rat model.* However, the rat does not express PP13and therefore one of us (George Osol) and his group are using the lantile virus model to examine this aspect. 

Is the DelT_221_ mutant less pro-inflammatory than the wildtype PP13? A study by one of us (Berthold Huppertz) and his group is currently conducted to compare the utero-placental vasculature between PP13 and its truncated variant showing major differences in the level of angiogenesis.

The *u*NK cells were shown to play a significant role in spiral artery remodeling [37]. Infect, it was shown that PP13 impact this process by inducing the release of IL-6 and IL-1α from *u*NK cells [19]. Our group has already demonstrated that in rats the long term exposure to PP13 is associated with uterine artery vasodilation and angiogenesis. The integration of all these components in the rat model is awaiting further research.

### The study limitations

The study limitations derived from several origins: (1) The effect of PP13 in changing blood pressure and arterial expansion was not explored in a preeclampsia animal model. Such a study is a crucial next step. (2) The CRD mutation was so far identified only among black and colored women in Africa and its importance as a factor in the development of preeclampsia among other ethnic groups was not yet established. The larger cohort explored now may shed light on the presence of the mutation elsewhere. (3) The PP13 molecule has additional domains that were not studied here. The heterogeneous nature of the syndrome of preeclampsia requires assessing the role of additional molecular domains of PP13 and exploring their relevance to preeclampsia in order to fully understand the role of PP13 in normal and impaired pregnancy.

### Conclusions

This study emphasizes the importance of truncated PP13 for the purpose of research in understanding the role of PP13 in blood vessels adaptation for pregnancy and placental development and preeclampsia. PP13 in animal blood causes a reduction in blood pressure as well as vascular expansion. We have no clear information as to what are the proteins to which PP13 in the blood is binding to but sugar residues of several proteins appear to be candidates for such interactions [10], [25]. Blood pressure regulation seems to be less demanding to having a CRD domain while arterial expansion seems to be much more dependent on the presence of the CRD molecular component. PP13 can be associated with several steps in normal and impaired development of the utero-placental vasculature and further research is required to complete our understanding of the involvement of reduced PP13 levels in the development of preeclampsia. Nonetheless, this study emphasizes that the CRD domain has multiple effect including immuno-tolerance [14], [19] and remodeling of the uteroplacental vasculature. While the first is most likely working on a direct cell to cell interaction in the placenta, the latter could be mediated by PP13 released from the placenta into the maternal vascular system and most likely working on the maternal endothelial layer from the maternal circulation side.
